The article "Peripheral Neuropathic Facial/Trigeminal Pain and RANTES/CCL5 in Jawbone Cavitation" was published in 2015. Journal: Evid Based Complement Alternat Med.

# Peripheral Neuropathic Facial/Trigeminal Pain and RANTES/CCL5 in Jawbone Cavitation

**DOI:** 10.1155/2015/582520

**Published:** 2015-06-11

**Authors:** Johann Lechner, Volker von Baehr

**Affiliations:** ^1^Clinic for Integrative Dentistry, Gruenwalder Strasse 10A, 81547 Munich, Germany; ^2^Medical Diagnostics-MVZ GbR, Nicolaistrasse 22, 12247 Berlin, Germany

## Abstract

*Introduction*. In this study, we elucidate the possible causative role of chronic subclinical inflammation in jawbone of patients with atypical facial pain (AFP) and trigeminal neuralgia (TRN) in the local overexpression of the chemokine regulated on activation and normal T-cell expressed and secreted (RANTES/C-C motif ligand 5 CCL5). Neurons contain opioid receptors that transmit antipain reactions in the peripheral and central nervous system. Proinflammatory chemokines like RANTES/CCL5 desensitize *μ*-opioid receptors in the periphery sensory neurons and it has been suggested that RANTES modifies the nociceptive reaction. *Materials and Methods*. In 15 patients with AFP/TRN, we examined fatty degenerated jawbone (FDOJ) samples for the expression of seven cytokines by multiplex analysis and compared these results with healthy jawbones. *Results*. Each of these medullary jawbone samples exhibited RANTES as the only highly overexpressed cytokine. The FDOJ cohort with AFP/TRN showed a mean 30-fold overexpression of RANTES compared to healthy jawbones. *Conclusions*. To the best of our knowledge, no other research has identified RANTES overexpression in silent inflamed jawbones as a possible cause for AFP/TRN. Thus, we hypothesize that the surgical clearing of FDOJ might diminish RANTES signaling pathways in neurons and contribute to resolving chronic neurological pain in AFP/TRN patients.

## 1. Introduction

The etiology of chronic facial pain is challenging to diagnose and difficult or frustrating to treat. Many different concepts have been presented and discussed, for example, the presence of a neuroma, implying that the nerve has been damaged in the periphery, and intracranial vascular compression of the trigeminal nerve root at the base of the skull. In 1997, Jannetta published a long-term follow-up study of the surgical approach to move the superior cerebellar artery away from the nerve root, maintaining the artery in its new position with a suture [1]. Various complementary various medical treatments for this problem, such as use of carbamazepine, have been reported [2]. Chronic facial pain can also be related to the temporomandibular joint (TMJ) and can be due to involvement of the cervical plexus [3]. Different terms have been used to describe atypical facial pain (AFP) such as atypical odontalgia (AO, also known phantom tooth pain), psychogenic toothache, and persistent dentoalveolar pain disorder [4]. International associations for the study of pain have adopted the term “persistent idiopathic facial pain” (PIFP) to replace AFP [5]. Pain is also one of the hallmarks of inflammation. Acute trigeminal pain is unavoidable given our interaction with dental decay, but it is just the tip of a disease iceberg. Below the surface of acute bacterial or viral infections lie chronic inflammations, the products of an immune system that is being constantly triggered by overexpressed cytokines. These triggers lead to the stimulation of different signaling pathways, which are instrumental in the development of chronic or “silent” inflammation. The signal messengers, such as the cytokines, carry instructions that are received by cells with specific receptors, which are able to detect them. Most dental procedures consist in eliminating acute inflammation in situations that do not feature typical signs of inflammation like pain and tissue swelling. This is the case with root fillings and surgical procedures like wisdom tooth surgery. The use of antibiotics helps the dentist and the patient overcome inflammation after dental procedures and during acute infections in daily practice. In daily dental practice, the effects of chronic inflammation on overall health are normally not of interest because local problems seem to be resolved after the symptoms of acute inflammation are gone. Consequently the individually targeted diagnosis of chronic pain in the peripheral facial nerves is a mostly neglected item in normal dental praxis even though this sensory disturbance in particular has a strong negative impact on the quality of life of those who are affected. Peripheral nerves are the source of almost all forms of neuropathic pain. Neuropathic pain is a complex syndrome resulting from many different forms of peripheral nerve damage, such as traumatic nerve damage, diabetes, and infections, as well as immune system and metabolic diseases [6]. For decades, a neuron-centered argument has been frequently used to explain the pathophysiology of chronic pain; however, recent studies have shifted attention towards a neuroimmune interaction. The concept of perineural jawbone inflammation producing or inducing facial neuralgias is an old one, and many oral surgical procedures have been recommended for “*tic douloureux*” [7]. This line of reasoning shifted when, in 1992,* Bouquot* examined 224 tissue samples from the mandibular alveolar bone of 135 patients with AFP or trigeminal neuralgia (TRN). All samples showed the clear presence of fatty-degenerative osteonecrosis spreading up to several centimeters in the form of retromolar cavities in the cancellous bone. This brought* Bouquot* to propose the term “*Neuralgia-Inducing Cavitational Osteonecrosis (NICO)*” to describe the clinical phenomenon of neuralgia in conjunction with fatty-degenerative osteolysis and osteonecrosis of the jawbone (FDOJ) [8]. Further reports in the dental literature suggest that curettage of jawbone lesions is an effective treatment for the pain associated with avascular FDOJ [9, 10]. Notwithstanding these reports, the underlying effects of FDOJ on AFP/TRN remain unexplored by modern immunological means. In contrast to former destructive, intracranial, and extracranial ablative approaches to branches of the trigeminal nerve our hypothesis is that the reduction of acute inflammation might serve as the beginning of a possible development of chronic inflammation in jawbone. Persons with certain risk factors might be prone to developing subsequent chronic AFP/TRN. Although a multidisciplinary approach is required to address the many facets of this pain syndrome, no studies of AFP/TRN have established a connection between the direct role that cytokines and chemokines play in the pain-affected area or in pain syndromes of the jawbone. Elucidating the mechanisms, defining successful treatment strategies and a critical attitude to operation sites with insufficient wound healing in jawbone and treatments tailored to AFP/TRN is a crucial part of the here-presented therapeutic concept.

## 2. Materials and Methods

### 2.1. Patient Cohort

This study was performed as a randomized controlled trial. We collected FDOJ tissue samples from 15 patients with AFP/TRN. A diagnosis of AFP/TRN was made by neurologists, pain specialists, and physicians. Inclusion criteria were (1) therapy-resistant pain that was clinically similar to AFP/TNR and (2) the local diagnosis of FDOJ in the painful jaw site. Mandatory inclusion criteria were (3) the availability of two-dimensional orthopantomograms (2D-OPG) and (4) cone beam three-dimensional (digital volume tomograms DVT) images. A further inclusion criterion for the group with surgery in the AFP/TRN areas was the measurement of bone density of the jawbone with transalveolar ultrasound technology (TAU). Besides 2D-OPG and 3D-DVT, the definite indication for FDOJ surgery was the additional measurement of bone density by TAU. TAU is a useful tool for establishing FDOJ [11–13]. Patients taking any medications due to neuropathic complaints were not excluded from the study. Demographic data from the AFP/TRN cohort showed an average age of 60 years (standard deviation (SD) = 13.2 years) and a gender ratio of 14 : 1 (female : male). The age range of the control group of 19 patients without FDOJ extended from 38 to 71 with an average age of 54 years and a gender split (female : male) of 11/8. This research was based on data retrieved from patients during normal dental surgery. All patients provided written informed consent.

### 2.2. Clinical Features of FDOJ Samples

The softening in FDOJ bone marrow is so distinct that the marrow space can be sucked and spooned out. Hollow cavitations with fatty degenerated adipocytes have undergone dystrophic changes accompanied by demyelination of the bony sheath of the infra-alveolar nerve. All 15 FDOJ samples presented clinically and macroscopically as fatty lumps. FDOJ is similar to silent inflammation or subclinical inflammation without the typical signs of acute inflammation.  Figure 1 shows a specimen with predominantly fatty transformation of the jawbone (a). The often-impressive extent of FDOJ lesions is illustrated in the right-hand panel by an X-ray with contrast medium.

### 2.3. Sampling of FDOJ Tissue

The current treatment of FDOJ lesions consists of curettage of the bony cavity, which relieves symptoms of pain with varying rates of success [8, 10, 14, 15]. To elucidate a possible causative link between FDOJ and AFP/TRN at the Munich Clinic for Integrative Dentistry, Germany, 15 patients with AFP/TRN and who were diagnosed with FDOJ had surgery on the affected area of the jaw. After local anesthesia and folding of a mucoperiosteal flap, the cortical layer was removed. All 15 patients exhibited FDOJ inside the bone marrow, which was quite similar to the samples described in the literature [8, 10]. In all 15 cases, surgery was performed on edentulous jaw areas in the sites of former wisdom teeth and the adjacent retro molar areas. The FDOJ samples, with a volume of up to 0.5 cm³, were stored in dry, sterile, 2 mL collecting vials (Sarstedt AG and Co, Nümbrecht, Germany), which were airtight, and frozen at −20°C. In addition to the cytokine analysis, we checked the FDOJ samples for pathohistological findings.

### 2.4. Processing of Necrotic Tissue Samples and Cytokine Measurements

In the examining Institute for Medical Diagnostics, Nicolaistrasse 22, 12247 Berlin inspected by DAKKS (Deutsche Akkreditierungsstelle GmbH, accredited to DIN EN ISO/IEC 17025:2005 and DIN EN ISO 15189:2007), the samples were homogenized by mechanical force in 200 *μ*L of cold protease inhibitor buffer (Complete Mini Protease Inhibitor Cocktail; Roche Diagnostics GmbH, Penzberg, Germany). The homogenate was then centrifuged for 15 minutes at 13,400 rpm. Next, the supernatant was collected and centrifuged for further 25 minutes at 13,400 rpm. In the 15 supernatants of tissue homogenate, we measured, regulated on activation, normal T-cell expressed and secreted (RANTES), also known as chemokine C-C motif ligand 5 (CCL5), FGF-2, interleukin- (IL-) 1 receptor antagonist (ra), IL-6, IL-8, monocyte chemotactic protein-1 (MCP1), and tumor necrosis factor-alpha (TNF-*α*). Measurement was performed using the Human Cytokine/Chemokine Panel I (MPXHCYTO-60K; Merck KGaA, Darmstadt, Germany) according to the manufacturer's instructions and analyzed using Luminex 200 with xPonent software (Luminex Co, Austin, TX, USA).

### 2.5. Pathohistological Examination

Parallel to the cytokine analysis, each FDOJ sample was examined histopathologically (Institute for Pathology & Cytology; Drs. Zwicknagel/Assmus, 85635 Freising, Germany).

## 3. Results

As we showed in earlier publications [15, 16], the defining feature of the FDOJ areas is overexpression of the proinflammatory messenger RANTES, also known as CCL5. The results of the multiplex analysis of the seven cytokines in the AFP/TRN cohort (*n* = 15) are shown in Table 1: AFP/TRN patients show elevated inflammatory signals in the FDOJ samples, deriving from painful jawbone areas with an average RANTES/CCL5 value of 4.274,7 pg/mL (SD = 2.778 pg/mL), compared to the randomized controlled sample of 149.9 (pg/mL) in healthy jawbone (Figure 2). All other cytokines were not derailed; only FGF-2 (fibroblast growth factor 2) and IL-1ra (interleukin 1 receptor antagonist) were additionally slightly upregulated in FJOD samples.

In the pathohistological findings the amount of fat cells was consistently and strikingly increased in FDOJ samples. Typical signs of inflammation, especially of an inflammatory cell response, were absent. The fatty-degenerative and osteolytic aspects occurred due to insufficient metabolic supply in an ischemic state. The histologic examination of the curetted tissue demonstrated ischemia (*n* = 13), necrotic adipocytes (*n* = 10), myxoid degeneration (*n* = 12), and increased fat cells (*n* = 12); inflammatory cells were only found in one FDOJ sample. Table 1 shows the pathohistological findings in FDOJ samples from 15 patients with AFP/TRN.

## 4. Discussion

### 4.1. Histology in Neuropathic Facial Pain

The presence of inflammatory cells in only one FDOJ sample confirms inflammation-free progression and the absence of inflammatory granulation in FDOJ [17, 18]. This raises an important question: Are typical infections the underlying cause of chronic AFP/TRN? In summary, the pathohistological findings clearly show that AFP/TRN is not caused by an osteitic process that might produce typical symptoms like swelling and local inflammation; this is the likely reason why former attempts to diminish AFP/TRN by serial extraction of apical inflamed teeth exhibited poor success. In these cases, the alveolar jawbone remained untouched and the “silent inflammation” in the affected area continued unabated. FDOJ must not be lumped together with other forms of osteomyelitis, which are defined by a dramatic increase in inflammatory cells.

### 4.2. Hyperactivated Chemokine RANTES/CCL5 in FDOJ

The absence of acute inflammation in FDOJ indicates that these chronic immunological processes are under the guidance of RANTES/CCL5, a proinflammatory chemokine. The hypothesis that FDOJ is an insidious, subtle process is supported by the fact that typical acute inflammatory cytokines, such as TNF-*α* and IL-6, were not increased in our samples. Proinflammatory cytokines have been repeatedly associated with demyelination and degeneration of the peripheral nerves, increased excitability of sensory afferents, and the induction of neuropathic pain [19]. The significance of RANTES to the development of disease appears to be substantial: RANTES interferes with immune responses on a number of levels and therefore plays a crucial role in pathological states. The chemotactic properties of RANTES send T-cells, dendritic cells, eosinophils, natural killer (NK) cells, mast cells, and basophils to the sites of inflammation and infection [20]. RANTES is also an effective activator of leukocytes, which play a key role in a wide range of inflammatory disorders [21], including in rheumatoid arthritis [22] and diseases of the central nervous system, such as multiple sclerosis [23]. RANTES has also been associated with the induction or promotion of cancer [24]. RANTES levels were markedly elevated in the primary tumor and metastatic lesions of all patients with breast and cervical cancer in a previous study [25].

### 4.3. Origin of RANTES in FDOJ—Fatty Tissue and Adipocytes

Reduced blood flow and capillary density followed by ischemia may lead to a hypoxic environment [26]. Moreover, adipocytes and necrotic fat cells are considered immunologically effective ingredients. For instance, Huber et al. found increased expression of RANTES in fatty tissue in obese patients [27]. The role of these immune effects in understanding FDOJ, RANTES/CCL5, and facial pain is an evident issue that will be further illuminated later in the discussion.

### 4.4. Immunology in Neuropathic Facial Pain

Recent data suggest that there is a strong link between immune and glial cells and the development of neuropathic pain [19]. The present paper and other researches provide evidence that the nearly 30-fold overexpression of chemokine RANTES/CCL5 that we found in the painful jawbone areas of the AFP/TRN cohort is linked to the disease development. Interactions between the immune and nervous systems occur at multiple levels, at which different types of immunologically active substances are involved in different stages of disease development [28]. Chronic pain is also associated with changes in neuroplasticity or changes in the neural pathways and synapses due to a defective reorganization of both the peripheral and central nervous systems. During tissue destruction, noxious stimuli and inflammation cause an increase in nociceptive input from the periphery to the central nervous system. Extended nociception from the periphery triggers a neuroplastic response at the cortical level and leads to a change in the somatotopic organization in the area of the body affected by pain; this results in central sensitization [19]. Moreover, immune activation near or around the peripheral nerves can cause increased excitability of these peripheral nerves. Both infectious substances and proinflammatory mediators may lead to changes in the blood-brain barrier (BBB) in response to chemotactic molecules that are released to the location of the damaged peripheral nerves which, in turn, leads neutrophils and macrophages to pass from the bloodstream into the nerves. Proinflammatory cytokines take part in this immune activation and shape the early immune response. However, these inflammatory mediators can directly increase nerve excitability, and they can cause damage to myelin and alter the permeability of the BBB. Furthermore, they can simultaneously lead to edema and further infiltration of the immune cells in peripheral nerves. Schwann cells, which ensheath the peripheral nerves, behave in a similar way to macrophages in the sense that they can present “non-self” substances to T-lymphocytes for further activation of immune cells. Schwann cells are also involved in the degradation of damaged myelin and cell debris [29]. Inflammatory mediators from the cells of the dorsal root ganglia (DRG), and those originating in the infiltrating immune cells and activated spinal microglia, are key elements that carry signal transmission of the pain response [10].

### 4.5. RANTES/CCL5 and Neuropathic Pain Syndromes

Cytokine/chemokine communication between glial cells and neurons is important for the development of neuropathic pain [30]. Studies indicate that prolonged chemokine and chemokine receptor activation in the sensory ganglia can significantly contribute to neuropathic pain syndromes. Long-term chemokine inflow through RANTES/CCL5 causes neuronal hyper excitability. While proinflammatory cytokines, such as TNF-*α*, IL-6, and prostaglandins, are already distributed early in the acute stage of an injury or tissue infection, there are many indications that chemokines are activated at a later time, and they can act in the conversion of acute pain into a more chronic phenomenon. Recent data suggest that, in conjunction with tissue damage or infection, ischemia-induced chemokine expression causes an increase in inflammatory cytokines and thus leads to the hyper excitability of sensory neurons [31]. Since some chemokine receptors, such as CCR2, CCR5, CXCR4, and CX3CR1, are located mostly in the primary afferent neurons or secondary neurons of the dorsal spinal horn [32], their chemokine ligands may be able to alter the quality of pain transmission. By means of peripheral administration of the chemokines CCL2, CCL3, CCL5, and CXCL12, it is possible to detect pain patterns that are caused by the activation of chemokine receptors in dorsal root ganglia [33]. A study that examined the effects of CCR5 deficiency on pain responses by employing CCR5 knockout (KO) mice found that the pain responses of CCR5 KO mice to chemical or inflammatory stimuli were milder than those of CCR5 wild-type mice [34]. Another study examined the effects of CCR5 deficiency on pain responses via the use of CCR5 KO mice; it was observed that the pain responses of CCR5 KO mice to chemical or inflammatory stimuli were milder than those of the CCR5 wild-type mice [33].

### 4.6. Opioid Receptors and Chemokine RANTES/CCL5

Recent studies have suggested that the chemokine RANTES and its receptor CCR5 interact directly with the opioid receptors and modify the nociceptive reaction [29]. Opioid receptors mediate antipain reactions, both in the peripheral and central nervous systems. The analgesic mechanism of morphine occurs when the analgesic opioid (e.g., morphine) excites the opioid receptors located in the brain and spinal cord; the perception of pain is blocked due to an agonistic, opposing effect. Morphine exerts its pain-relieving effect by binding to the nerve cells at the same binding sites as the endorphins; the specific binding sites are the opioid receptors. Fewer nociceptive neurotransmitters are released through morphine-induced opioid receptor excitation, and an incoming pain signal is not propagated. Studies have shown that opioid use suppresses chemokine-mediated chemotactic responses effectively, and this can be seen as a result of heterologous desensitization between opioids and some of the chemokine receptors [34]. The desensitization of opioid receptors through RANTES/CCL5 is part of this mutual “crossover” desensitization [35]. More recently, there have been reports showing that the process of heterologous desensitization is bidirectional, and that chemokine receptor activation leads to an inactivation of the in vitro activity of opioid receptors [36]. An open question that remains is whether some chemokines have the ability to desensitize opioid receptors in vivo. Studies using a rat model found that the analgesic response was blocked in opioids following chemokine application [37, 38]. In these studies, Pizziketti et al. were able to show that proinflammatory chemokines, such as CCL2/MCP-1, CCL5/RANTES, and CXCL8, are able to desensitize *μ*-opioid receptors on the peripheral sensory neurons [39]. Therefore, these *μ*-opioid receptors offer novel and potential mechanisms for peripheral inflammation-induced hyperalgesia. Scientists believe that this neural overexcitation materializes during chronic exposure to RANTES/CCL5 through the local overexpression in all trigeminal cases within the FDOJ and thus inhibits RANTES activity on the *μ*-opioid receptors in the synapses. Moreover, chemokine-induced desensitization is mediated by the chemokine receptors [40]. Animals directly injected with specific doses of RANTES/CCL5 in the periaqueductal gray matter, a brain region that is the first to handle the antinociceptive effects of opioids, experience blocked and altered normal pain response to opioids. Our data indicate that proinflammatory chemokines are capable of desensitizing *μ*-opioid receptors on peripheral sensory neurons, providing a novel potential mechanism for peripheral inflammation-induced hyperalgesia [40]. When the interval of the chemokine effect was extended to 2 hours, the ability of RANTES/CCL5 to desensitize opioid receptors was lost. A logical explanation for this is that the desensitization of opioid receptors is a reversible process that occurs via metabolic degradation. In our clinical neuralgia cases, the hypothesis of RANTES/CCL5 as a source of pain has persisted for years, so the experimental time limit for RANTES/CCL5 exposure on the opioid receptors is irrelevant. The above-cited experiments show that the opioid receptors can be desensitized by treatment with chemokines, which suggests that the desensitization of all three opioid receptors is achieved through the activation of RANTES/CCL5 [36]. Although RANTES/CCL5 desensitizes opioid receptors very effectively, desensitization does not work with all chemokines [41]. Recent studies have also shown that the chemokine/RANTES receptor CCR5 interacts with opioid receptors and leads to a change in the nociceptive reaction [42].

### 4.7. Diagnostic Problems of FDOJ Lesions by X-Ray

The nonvisible nature and lack of radiographic appearance of FDOJ make it difficult to obtain an accurate diagnosis [13]. Therefore, the existence of FDOJ is largely neglected today in mainstream dentistry. The reason for this is that conventional X-ray techniques are limited in their ability to reveal the actual extent and location of FDOJs. To aid the practitioner in diagnosing the debilitating effects of bone marrow softening inside FDOJ lesions, a computer-assisted TAU device was developed [43]. TAU precisely images and identifies cavitational porosity in the jawbone. Studies show that, in 84% of cases, FDOJ lesions on TAU images were more obvious and more readily identified than on radiographs of the same site. TAU imaging proved to be significantly superior to radiology for the detection of microscopically confirmed FDOJ. The efficiency and reliability of TAU in the diagnosis and imaging of FDOJ have been presented in earlier publications [44]. Because of these diagnostic difficulties, FDOJ as a presumably widespread jawbone disease is underdiagnosed by dentists in general; specifically, in AFP/TRN cases, it may often falsely be referred to as “idiopathic.”

The clinical example in Figure 3(a) shows the typical situation during surgical debridement and curettage of the lower jaw. The infra-alveolar nerve is totally denuded from its bony sheath by FDOJ. The ischemic process of FDOJ converts the bony sheath, leaving the nerve tissue intact. As evidenced by what is not shown in the X-ray in the right-hand panel of the figure, this process is inconspicuous and does not show any signs of inflammation or FDOJ. Because of this diagnostic problem of identifying FDOJ on common dental X-rays [13], this patient suffered from AFP for 7 years and received antidepressants during this time as a singular therapy.

### 4.8. Clinical Relevance of FDOJ Surgery in AFP/TRN Cases

The neurological theories and the data we retrieved from the FDOJ surgery resulted in pain relief in our AFP/TRN cohort. The subjective pain intensity in our AFP/TRN cohort was measured using the Numeric Rating Scale (NRS) [45]. The results of the NRS (ranging from 1 to 10) were changed into a percentage to evaluate pain relief.  Figure 4 shows the mean time of AFP/TRN (45 months), the pain-free period after FDOJ curettage (21 months at the time the statistic was measured), and the overall percentage of pain relief (88%) in our 15 patients. Details of pain reduction in each patient are shown in Figure 5, which documents a mean percentage of 88%. Similar results in AFP/TRN pain relief were reported in other papers discussing FDOJ curettage [46].

### 4.9. A Clinical Case of FDOJ Surgery (Figure 6)

To show the extent to which curettage of FDOJ in patients affected by AFP/TRN can contribute to alleviating facial pain and to give an example of the clinical relevance of FDOJ, our patient Mrs. N. T. reported the following: “*Since spring 2009 I had been getting recurring stabbing pain on the left-hand side of my face and earache, tinnitus and pain in my shoulder/arm. During the night I suffered palpitations and panic attacks. My physical energy levels also dropped. I consulted a further two dentists to no avail. One recommended that I went to see a neurologist, who prescribed me strong painkillers and psychotropic drugs. A trip to an osteopath was also unfortunately fruitless. In summer 2011 I was in a horrendous amount of pain, particularly at night. I could barely sleep through the night. I was taking strong painkillers every day just to get me to work. Then came the day when everything was solved. On 15 February 2012 I had an operation on the left side of my upper jaw and bone was excavated. After about 4 weeks I was almost pain-free without medication*.”

## 5. Conclusions

Although the role of proinflammatory cytokines and chemokines has been identified in neuropathic pain [38], the exact relationship between the chemokine–cytokine network and neuropathic pain is not fully understood. Jawbone cavitations are hollow dead spaces in the jaw bone, where the bone marrow is dying or dead. The research suggests that this jawbone disease, known popularly as “cavitations” and in some technical publications as “NICO,” might serve as a fundamental cause of neuropathic pain, through the inflammatory cytokines that it produces. Opioid receptors mediate antipain responses in both the peripheral and central nervous systems, and RANTES/CCL5 is able to enhance the pain response. As RANTES/CCL5 is overexpressed in jawbone areas defined by FDOJ, this process close to the trigeminal nerve might contribute to the development of AFP/TRN. Data from our research points to the local overexpression of RANTES/CCL5 in jawbones as a possible additional cause of AFP/TRN. Treatment for more advanced stages of FDOJ requires surgery. Surgical debridement of FDOJ areas can diminish RANTES/CCL5 overexpression and thus reduce chronic facial pain. The success of such surgery is by no means guaranteed and it depends on the technique and the skill of the dentist doing the surgery. FDOJ, as a contributing factor to AFP/TRN, is a widely neglected form of “silent inflammation” characterized by the overexpressed chemokine RANTES/CCL5. When doctors or dentists are presented with AFP/TRN of undetermined origin or that is “idiopathic,” a complete differential diagnosis should include FDOJ lesions. The presence of FDOJ is often not entirely obvious from examination of a panorex or other X-rays. Many case histories in our clinic show that removing the diseased FDOJ from the jawbone may be the key to reversing the course of different forms of AFP/TRN. Further studies are needed to fully understand the neuropathic regulatory mechanisms that underlie neuroinflammation following nerve damage by cytokines deriving from FDOJ.

## Figures and Tables

**Figure 1:** FDOJ sample of fatty and osteolytic degenerated bone marrow (a) and contrast medium X-ray of the FDOJ cavity after curettage (b).

**Figure 2:** Analysis of seven cytokines in the FDOJ AFP/TRN cohort (*n* = 15) compared to healthy jawbones.

**Figure 3:** Curettage of FDOJ in the lower jaw with denuded infra-alveolar nerve. Corresponding X-ray without any signs of pathological process in jawbone (b).

**Figure 4:** Mean time of AFP/TRN (45 months), the pain-free period after FDOJ curettage (21 months), and the overall percentage of pain relief (88%).

**Figure 5:** Percentage of pain reduction in the AFP/TRN cohort (*n* = 15).

**Figure 6:** A patient with AFP in the left upper jaw with overexpression of RANTES/CCL5 in the painful area. The corresponding X-ray marked in red is inconspicuous; pain relief after FDOJ surgery was 90%.

**Table 1:** Pathohistological findings from FDOJ samples in 15 patients with AFP/TRN.

AFP/TRN	15	100%
Ischemia	13	87%
Necrotic adipocytes	10	67%
Myxoid degeneration	12	80%
Increased fat cells	12	80%
Inflammatory cells	1	7%
